# Relationships of Serum Homocysteine, Vitamin B_12_, and Folic Acid Levels with Papulopustular Rosacea Severity: A Case-Control Study

**DOI:** 10.1155/2022/5479626

**Published:** 2022-07-04

**Authors:** Bo Young Chung, Hye One Kim, Chun Wook Park, Na Gyeong Yang, Jae Yun Kim, Yun Su Eun, Euy Hyun Chung, Sung Yul Lee, Young Lip Park, Sang Hoon Lee, Nam Hun Heo, Min Jeong Shin, Jung Eun Kim

**Affiliations:** ^1^Department of Dermatology, Hallym University Kangnam Sacred Heart Hospital, Hallym University College of Medicine, Seoul 07441, Republic of Korea; ^2^Department of Dermatology, Soonchunhyang University Cheonan Hospital, Soonchunhyang University College of Medicine, Cheonan 31151, Republic of Korea; ^3^Department of Dermatology, Soonchunhyang University Bucheon Hospital, Soonchunhyang University College of Medicine, Bucheon 14584, Republic of Korea; ^4^Soonchunhyang University Hospital Cheonan, Clinical Trial Center, Republic of Korea; ^5^Soonchunhyang University Graduate School of Medicine, Asan 31538, Republic of Korea

## Abstract

**Background:**

Rosacea is a chronic inflammatory skin disease with a multifactorial etiology. Recently, associations between serum homocysteine (Hcy) levels and inflammatory skin diseases, such as psoriasis and hidradenitis suppurativa, have been reported. However, no study has explored the levels of serum Hcy, folic acid, and vitamin B_12_ in patients with rosacea.

**Objective:**

To investigate serum Hcy, vitamin B_12_, and folic acid levels in patients with papulopustular rosacea (PPR), we characterized the association of these levels with PPR severity.

**Methods:**

This case-control study included 138 PPR patients and 58 healthy controls. The serum levels of Hcy, vitamin B_12_, and folic acid were measured. A correlation was assessed between disease severity and serum levels of Hcy, vitamin B_12_, and folic acid.

**Results:**

Serum vitamin B_12_ and folic acid levels were significantly lower in PPR patients than in the healthy controls (*p* = 0.011 and *p* = 0.0173, respectively). Although serum Hcy levels did not significantly differ between PPR patients and healthy controls, PPR severity was positively correlated with serum Hcy levels (*p* < 0.001).

**Conclusions:**

Our results suggest a possible association between hyperhomocysteinemia and vitamin B_12_ deficiency in patients with PPR.

## 1. Introduction

Rosacea is a chronic inflammatory skin disease that occurs frequently in women and individuals with fair skin [1]. The disease is characterized by recurrent flushing, erythema, papules, telangiectasia, edema, pustules, or a combination of these symptoms with an uncertain etiology [2]. Clinically, rosacea can be categorized into four subtypes based on the predominant signs and symptoms: erythematotelangiectatic, papulopustular, phymatous, and ocular [3]. The protracted disease course, tendency for recurrence, facial complexion-related changes, skin ulceration, and scar formation in rosacea tend to have detrimental effects on the physical, mental, and social health of affected patients [4]. The exact pathophysiology of rosacea is not fully understood, but genetic factors, immune dysregulation, microorganisms, chronic inflammation, vascular hyperreactivity, and other environmental factors are considered to play a role in its development [5–8]. Recent studies have shown that reactive oxygen species (ROS) are related to inflammation in rosacea [9, 10].

Chronic inflammation plays a pivotal role in the pathogenesis of rosacea. Dysregulation of the immune system, vascular changes, and oxidative tissue damage are the factors associated with the inflammation of rosacea [7, 11, 12]. Oxidative stress is a pathological state caused by the disequilibrium between oxidants and antioxidants. Increased ROS levels may promote inflammation by activating multiprotein cytoplasmic complexes called inflammasomes [13, 14]. As a result, increased levels of proinflammatory cytokines may damage various cells, including endothelial cells, keratinocytes, and fibroblasts.

Hcy is a sulfur-containing amino acid generated as a result of the metabolism of methionine. Hcy is converted to methionine or cystathionine, with vitamin B_12_ and folate as cofactors. In the metabolic cycle of Hcy synthesis, deficiencies in these vitamin-containing cofactors lead to higher levels of Hcy and lower levels of methionine [15, 16]. Hyperhomocysteinemia is associated with various systemic diseases, including cardiovascular, cerebrovascular, and neuropsychiatric conditions [17–19]. Several studies have revealed multiple potential mechanisms by which homocysteine (Hcy) may contribute to the development of endothelial dysfunction and atherosclerosis, including platelet activation and oxidative stress [20–23]. Many studies have demonstrated an increased incidence of hyperhomocysteinemia in patients with various inflammatory skin diseases, including acne, vitiligo, psoriasis, and hidradenitis suppurativa [24–27]. However, to the best of our knowledge, no study has explored the serum levels of Hcy, folic acid, and vitamin B_12_ in patients with rosacea. Thus, this study is aimed at analyzing serum Hcy, vitamin B_12_, and folic acid levels in patients with papulopustular rosacea (PPR) and then characterized the associations of these levels with PPR severity.

## 2. Materials and Methods

### 2.1. Ethical Considerations

This prospective, case-control study was approved by the Institutional Review Boards (IRBs) of Soonchunhyang University Cheonan Hospital (IRB number: 2018-07-059) and Hallym University Kangnam Sacred Heart Hospital (IRB number: 2019-07-011). This study was designed and performed in accordance with the framework and ethical guidelines of the Declaration of Helsinki. Informed consent was obtained from all participants.

### 2.2. Patients

A total 196 participants were included in the study, including 138 newly diagnosed treatment-naïve PPR patients and 58 healthy controls. Rosacea severity was assessed using the National Rosacea Society grading system. In addition, the patients were recommended to self-assess their skin lesions and label them as 1 = mild, 2 = moderate, and 3 = severe. Clinical and laboratory variables were reviewed and analyzed. The patients included in the study were aged ≥18 years and had newly diagnosed treatment-naïve PPR. Exclusion criteria included a history of a cardiovascular event; body mass index (BMI) > 30; an abnormal increase in transaminase levels; presence of diabetes mellitus, hypertension, chronic kidney or liver disease, neuroendocrine disorders, malignancy, serious infectious disease, or another concomitant inflammatory or metabolic condition; a history of using medication with effects on serum Hcy, folate, and vitamin B_12_ levels (e.g., phenytoin, carbamazepine, penicillamine, theophylline, vitamins, folate, oral contraceptive pills, azathioprine, metformin, thiazide diuretics, isotretinoin, and antibiotics) for at least three months prior to the study; presence of psoriasis; and a history of cigarette smoking. Healthy controls were comprised of age- and sex-matched healthy individuals who attended the hospital for routine medical examinations. Pregnant and lactating women were excluded from both groups.

### 2.3. Estimation of Hcy, Vitamin B_12_, and Folic Acid Levels

Venous blood samples (4 ml) were collected from participants in both groups. Before analysis, the samples were immediately centrifuged and stored at -80°C. The total serum Hcy levels were measured using a Cobas 8000 c702 analyzer (Roche Diagnostics, Mannheim, Germany). The serum levels of vitamin B_12_ and folic acid were measured using a Cobas 8000 e801 analyzer (Roche Diagnostics).

### 2.4. Measurements of TEWL, Skin Hydration, and Demodex Mite Density

Transepidermal water loss (TEWL, g/h/m^2^) was measured using a VapoMeter (Delfin Technologies, Kuopio, Finland), and skin hydration (arbitrary units) was measured using a Moisture MeterSC Compact (Delfin Technologies). The measurement devices were placed on the cheek skin at lesion sites and were held vertical to the skin surface in accordance with the manufacturer's recommendations. The measurements were performed three times, within two minutes of each other, and the mean values were recorded. All measurements were conducted in a room that was not controlled by the climate. The temperature and humidity in the room were generally stable (20–24°C and 40–60% relative humidity). In addition, a standardized skin surface biopsy was performed to measure *Demodex* mite density. A standard area of 1 cm^2^ was drawn on a slide using a waterproof pen. A drop of cyanoacrylic adhesive was then placed on the other side of the slide, and the adhesive-bearing surface was applied to the skin for one minute. After the adhesive was allowed to dry, the slide was gently removed with the surface skin. The sample was clarified with one to two drops of immersion oil and covered with a coverslip. The samples were examined under an optical microscope (×40, ×100).

### 2.5. Statistical Analysis

All statistical analyses were performed using IBM SPSS Statistics for Windows, version 26.0 (IBM Corp., Armonk, N.Y., USA). Results are expressed as mean ± standard deviation. In all analyses, *p* < 0.05. One-way analysis of variance or the Kruskal-Wallis test was used for comparisons between more than two groups. The chi-square test was used to compare the differences in constituent ratios between PPR patients and healthy controls. Rosacea severity and serum homocysteine (Hcy), vitamin B_12_, and folate levels were analyzed using linear analysis.

## 3. Results

The current hospital-based case-control study included PPR patients (*n* = 138) and normal healthy controls (*n* = 58). The baseline clinical characteristics of the participants are presented in Table 1. Patients and controls were adequately matched, and there were no significant differences in the mean age, sex distribution, or body mass index between the two groups (*p* = 0.0976, *p* = 0.5535, and *p* = 0.2467, respectively). Serum levels of Hcy in PPR patients were 10.79 ± 2.96 and 10.15 ± 3.16 in healthy controls (*p* = 0.0671). However, serum vitamin B_12_ and folic acid levels were significantly lower in PPR patients than in healthy controls (*p* = 0.011 and *p* = 0.0173, respectively).

The severity of rosacea, assessed using the National Rosacea Society clinical grading system [28], ranged from mild to moderate. In PPR patients, the Hcy level significantly differed according to the severity of rosacea (*p* < 0.001). Serum Hcy levels were significantly higher in male than in female patients (*p* = 0.0017; Figure 1(a) and Table 2). Serum vitamin B_12_ and folic acid levels also correlated with rosacea severity (*p* < 0.001; Figures 1(b) and 1(c) and Table 2). Moreover, serum Hcy levels were inversely correlated with serum folic acid and vitamin B_12_ levels (*r* = −0.287, *p* < 0.001 and *r* = −0.263, *p* < 0.001; Figures 2 and 3). TEWL and *Demodex* density were measured in 65 of 138 PPR patients; both were positively correlated with disease severity (*r* = 0.3583, *p* < 0.001 and *r* = 0.4951, *p* < 0.001; Table 3). TEWL significantly correlated with serum Hcy and folic acid levels (*r* = 0.358, *p* = 0.0034 and *r* = 0.288, *p* = 0.0202; Figure 4). *Demodex* density also showed statistically significant correlations with serum Hcy, vitamin B_12_, and folic acid levels (*r* = 0.495, *p* < 0.001; *r* = 0.272, *p* = 0.0283; and *r* = 0.526, *p* < 0.001; Figure 5).

## 4. Discussion

Mounting evidence suggests that rosacea may be an outcome of systemic inflammation [29]. Recently, several studies have reported associations between rosacea and various systemic disorders, although causal relationships have not been clearly determined [30–32]. In particular, the greatest evidence is an increased incidence of dyslipidemia, hypertension, and cardiovascular diseases in patients [30–35]. Since systemic inflammation is associated with both cardiovascular disease and rosacea, the studies suggest the assessment of risk for cardiovascular disease in rosacea patient [36, 37].

Although we did not find differences in Hcy levels between PPR patients and healthy controls, we found that Hcy levels correlated with rosacea severity. The serum Hcy level in patients with severe rosacea exhibited mild elevation compared with healthy controls (13.09 ± 2.87). However, we found that serum vitamin B_12_ and folic acid levels were significantly downregulated in patients with PPR compared to healthy controls. The more severe the rosacea, the lower the levels of vitamin B_12_ and folic acid (*p* < 0.001). Moreover, we found the serum Hcy level was inversely correlated with serum vitamin B_12_ and folic acid levels that are involved in Hcy metabolism [38, 39]. Serum Hcy levels were significantly higher in male (12.08 ± 3.36) than in female patients (10.27 ± 2.62). This may have occurred because the rosacea severity was more severe among male patients than females. Severe rosacea (severity grade 3) was observed in only 26.5% of female patients compared to 52.5% of male patients. It can be thought that male patients tend to visit the hospital only when symptoms become more severe than female patients, but the evidence from our study on this is insufficient.

Hcy is an intermediate sulfur-containing amino acid product of the normal methionine metabolism. It can be recycled into methionine, mainly in the presence of cofactors such as folic acid and vitamin B_12_. In the remethylation and trans-sulfuration pathways of Hcy metabolism, deficiency or defective metabolism of folic acid, vitamin B_12_, or pyridoxine leads to elevated levels of plasma Hcy, which is known as hyperhomocysteinemia [15, 16]. Hyperhomocysteinemia and vitamin B_6_, vitamin B_12_, and folic acid deficiencies can be caused by a variety of nutritional and genetic factor [40]. Inflammatory cytokines and chemokines involved in chronic inflammatory diseases appear to be activated by Hcy through the redox-sensitive NF-*κ*B pathway following oxidative stress [41]. Several studies have also shown that proinflammatory cytokines, such as tumor necrosis factor-alpha (TNF-*α*) and interleukin-1*β* (IL-1*β*), are increased in endothelial cells, retinal cells, and microglia by hyperhomocysteinemia [41–43].

UV radiation, heat, spicy food, alcohol, stress, or microbes are known rosacea triggers that induce primary proinflammatory cytokines such as TNF-*α* and IL-1 family members [12]. TNF-*α* and IL-1*β* are known to induce the expression of a subset of proinflammatory chemokines (CXCL1, CXCL8, CCL20, and CCL27) in keratinocytes, implying a potential pathway for TH1 and TH17 cell recruitment as well as neutrophil recruitment in rosacea lesional skin [12]. In addition, previous studies have linked rosacea to an imbalanced gut microbiome [44–46]. Egeberg et al. showed that the prevalence of gastrointestinal disorders such as celiac disease, Crohn's disease, ulcerative colitis, small intestinal bacterial overgrowth, and irritable bowel syndrome was significantly higher among patients with rosacea than among controls [47]. These gastrointestinal diseases and dysbiosis may lead to the impaired absorption of folate and vitamin B_12_. This, in turn, may cause hyperhomocystemia in rosacea patients. Therefore, an increase in Hcy levels may affect the pathogenesis of rosacea through an increase in these proinflammatory responses.

Hyperhomocysteinemia is a known risk factor for stroke, coronary heart disease, and peripheral vascular diseases. The mechanisms of atherothrombosis caused by hyperhomocysteinemia include endothelial dysfunction, increased platelet turnover, enhanced platelet activation, hypercoagulability, upregulation of tissue factors, and oxidative stress [48–50]. Previous studies have shown that vitamin B_12_ and folic acid deficiencies are associated with atherothrombotic complications. Many studies have provided strong evidence regarding the role of Hcy as an independent risk factor for atherosclerotic vascular disorders [51, 52]. Our findings may explain the increased susceptibility to cardiovascular disease in patients with rosacea. However, larger prospective studies are needed to evaluate the role of Hcy in cardiovascular comorbidities in patients with rosacea.

In our study, TEWL and *Demodex* density also showed positive correlations with disease severity and were significantly associated with serum Hcy and folate levels. Skin barrier defects are correlated with greater skin disease severity, making the skin more susceptible to *Demodex* mite infection in patients with rosacea (particularly PPR) [53]. Similarly, *Demodex* may affect the skin barrier integrity and induce inflammatory changes in the dermis via the production of vasoactive substances. It may also contribute to rosacea pathogenesis by stimulating the innate immune system through mechanisms such as antimicrobial peptides, Toll-like receptors, and activating innate immune cells [53]. Previous studies have shown that the antigenic proteins of *Bacillus oleronius*, which were isolated from a *Demodex* mite in a patient with rosacea, cause neutrophilic accumulation and induce an inflammatory response in neutrophils [54, 55]. As a result, myeloperoxidase (MPO) levels are elevated and MPO-derived oxidation products overcome the cellular antioxidant defense mechanism and contribute to oxidative stress. Considering that the lethal effects of neutrophils on microorganisms are dependent upon the production of ROS, they can also affect systemic oxidative stress, and matrix metalloproteinase (MMP) levels can increase as a result of neutrophil degranulation [7]. Recent data suggests a strict one-to-one relationship involving immune activation, inflammation, and Hcy levels [56]. These data may aid in explaining the mechanism underlying the abovementioned high Hcy levels in PPR. However, further research is required to confirm the potential correlations between immune activation, oxidative stress, and Hcy levels.

This study was limited by the small sample size. The correlation between serum levels of Hcy and rosacea severity shown in this study is probably an indirect effect. Additional large prospective studies are needed to evaluate the role of Hcy in cardiovascular comorbidities in patients with rosacea. Moreover, we do not know whether severe PPR symptoms occurred first or hyperhomocystemia. Thus, further work should be dedicated to determining how Hcy contributes directly to the pathogenesis of PPR, since changes in these serum parameters are also thought to be involved together with individual predisposition and environmental triggers. In addition, prevention via folate and vitamin B_12_ supplementation for therapeutic effects in patients with rosacea should also be investigated. However, to our knowledge, this is the first study to examine serum levels of Hcy, vitamin B_12_, and folic acid in patients with rosacea.

## 5. Conclusion

In conclusion, we found a significant positive correlation between the severity of rosacea and serum Hcy levels. Furthermore, this study showed significant decreases in serum vitamin B_12_ and folic acid levels in patients with rosacea compared with healthy controls; these changes were correlated with PPR severity. Our findings imply that physicians should be aware of possible hyperhomocysteinemia in patients with severe PPR. Although further prospective studies are needed to confirm the effects of vitamin B_12_ or folate in rosacea treatment, we suggest that dietary supplementation with folic acid and antioxidant vitamins in severe rosacea patients with hyperhomocysteinemia may improve rosacea symptoms by reducing blood Hcy levels.

## Figures and Tables

**Figure 1:** (a) Serum homocysteine levels. (b) Serum vitamin B_12_ levels. (c) Serum folate levels.

**Figure 2:** Serum folic acid levels are inversely correlated with serum homocysteine levels (*r* = −0.287, *p* < 0.001).

**Figure 3:** Serum vitamin B_12_ levels are inversely correlated with serum homocysteine levels (*r* = −0.263, *p* < 0.001).

**Figure 4:** TEWL correlate directly with serum homocysteine and folate levels. TEWL: transepidermal water loss.

**Figure 5:** *Demodex* density correlate with serum homocysteine, vitamin B_12_, and folate levels.

**Table 1:** Baseline characteristics of PPR patients and controls.

Variables	Total (*n* = 196)	PPR (*n* = 138)	Healthy controls (*n* = 58)	*p* value
Sex				
Male (1)	60 (30.61%)	40 (28.99%)	20 (34.38%)	0.5535
Female (2)	136 (69.39%)	98 (71.01%)	38 (65.52%)	
Age	45.46 ± 13.98	44.46 ± 13.36	47.84 ± 15.22	0.0876
BMI	22.88 ± 2.87	22.73 ± 2.95	23.24 ± 2.68	0.2467
Homocysteine	10.6 ± 3.03	10.79 ± 2.96	10.15 ± 3.16	0.0671
Vitamin B_12_	712.67 ± 300.85	691.72 ± 306.1	762.53 ± 284.34	0.011
Folate	12.51 ± 4.21	12.18 ± 4.35	13.31 ± 3.76	0.0173

PPR: papulopustular rosacea; BMI: body mass index.

**Table 2:** Serum levels of Hcy, vitamin B_12_, and folic acid of PPR patients according to rosacea severity grade and sex.

Variables	*n*	Homocysteine		Vitamin B_12_		Folate	
		Mean ± SD	*p* value	Mean ± SD	*p* value	Mean ± SD	*p* value
Rosacea severity							
1	40	8.61 ± 1.85	<0.001	783.2 ± 383.24	<0.001	14.96 ± 4.7	<0.001
2	51	10.39 ± 2.18		746 ± 274.54		12.91 ± 3.8	
3	47	13.09 ± 2.87		554.96 ± 207.23		9.02 ± 2.11	
Sex							
Male (1)	40	12.08 ± 3.36	0.0017	660.12 ± 354.52	0.0641	11.64 ± 4.42	0.259
Female (2)	98	10.27 ± 2.62		704.61 ± 284.99		12.39 ± 4.32	

Hcy: homocysteine; PPR: papulopustular rosacea; SD: standard deviation.

**Table 3:** *Demodex* density, TEWL, and hydration of PPR patients according to rosacea severity grade and patients' self-assessment.

Variables	*n*	*Demodex*		TEWL		Hydration	
		Mean ± SD	*p* value	Mean ± SD	*p* value	Mean ± SD	*p* value
Rosacea severity							
1	27	0.52 ± 0.85	<0.001	19.31 ± 8.18	<0.001	14.96 ± 4.7	0.2486
2	20	1.55 ± 1.36		20.75 ± 10.95		12.91 ± 3.8	
3	18	6.89 ± 2.78		37.29 ± 7.82		9.02 ± 2.11	
Patient's self-assessment							
1	13	0.31 ± 0.63	<0.001	18.59 ± 9.38	0.002	65.43 ± 26.89	0.4978
2	21	1.71 ± 3.24		20.53 ± 9.99		74.95 ± 20.97	
3	31	4.16 ± 3.06		30.16 ± 11.81		75.42 ± 24.41	

TEWL: transepidermal water loss; PPR: papulopustular rosacea; SD: standard deviation.

## Data Availability

The data used to support the findings of this study are available from the corresponding author upon request.
